# Ethnobotanical study of Mandi Ahmad Abad, District Okara, Pakistan

This article has been retracted.

**DOI:** 10.1371/journal.pone.0265125

**Published:** 2022-04-07

**Authors:** Mubashrah Munir, Sehrish Sadia, Adnan Khan, Bakht Zareen Rahim, Brian Gagosh Nayyar, Khawaja Shafique Ahmad, Arshad Mahmood Khan, Ishrat Fatima, Rahmatullah Qureshi

**Affiliations:** 1 Department of Biological Sciences, University of Veterinary and Animal Sciences, Lahore, Pakistan; 2 Department of Botany, University of Balochistan, Quetta, Pakistan; 3 Department of Botany, University of Sialkot, Sialkot, Pakistan; 4 Department of Botany, University of Poonch, Rawalakot, Azad Jammu and Kashmir, Pakistan; 5 Govt. Hashmat Ali Islamia Associate College Rawalpindi, Punjab, Pakistan; 6 Department of Botany, Pir Mehr Ali Shah Arid Agriculture University Rawalpindi, Punjab, Pakistan; Mirpur University of Science and Technology, PAKISTAN

## Abstract

This study hypothesized that native people have unique traditional knowledge of plant resources in the rural areas and basic objective was the documentation of this valuable inheritance. Ethnobotanical data was collected from a remote rural area of Mandi Ahmad Abad, Union council number NA-144 Tehsil Depalpur District Okara, Pakistan. A total of 94 informants were randomly interviewed to collect data about local names of plant species, mode of administration, recipes and ailments, and ethnobotanical uses through semi-structured questionnaire, interviews and group discussion methods. The collected data was statistically analyzed by calculating use value (UV), frequency of citation (FC), relative frequency of citation (RFC), factor of informant consensus (FIC), family importance value, and relative importance (RI). This study is also compared with ethnobotanical literature by using Jaccard’s index (JI) for similarity analysis. A total of 126 species belonging to 52 families were documented. The Poaceae (13spp.), Leguminosae (12spp.), Solanaceae (10spp.) and Cucurbitaceae (10spp.) were dominant families. Highest used value (UV = 0.22) was obtained for *Azadirachta indica*. The minimum used value (UV) was showed by *Alhagi maurorum*, *Eclipta prostrata*, *Hibiscus rosa-sinensis*, *Solanum virginianum* and *Trianthema potulacastrum* (UV = 0.01). Hepatitis, stomach ulcer, bowel disorders, urinary problems, psoriasis, cancer, and leucoderma were the most treated ailments with ICF value of 1, followed by leucorrhea (ICF: 0.89), and vomiting (ICF: 0.86). The highest Jaccard’s similarity index value (JI = 0.329) showed that plant species reported in our study was more similar with Arid regions of Northern Punjab, Pakistan. This novel ethnobotanical report concluded that traditional knowledge about use of medicinal plants is decreasing due to allopathic medicines. Immediate steps should be taken for conservation and documentation of traditional knowledge of plants especially those having medicinal properties.

## Introduction

Ethnobotany is a branch of science that studies the use of plants by local peoples and how plants are used for food, timber, fuel, ornaments, and medicines. One of the purposes of ethnobotanical is to report, record, and conserve the indigenous knowledge of plants [1]. Modern ethnobotany is involving in knowledge of botany, taxonomy, biochemistry, geology, and medicine etc. [2]. Since antient times, people have been using plants local to their villages for medicinal and other purposes [3, 4]. Traditionally, ethnobotanical knowledge has been passed down orally from generation to generation [5]. Conventional ethno-veterinary knowledge is generally still passed on orally. To prevent the extinction of this knowledge it is important to document it and preserve it for future generations [6].

Traditional knowledge about plants in China can be traced back to about five thousand years. According to a report from the World Health Organization, almost eighty percent of the current population in developing countries still depends on the usage of traditional plant knowledge [7, 8]. The folk knowledge of indigenous plants plays an important role in the discoveries of many vital modern-day drugs. Almost 25% of drugs in modern medicines are obtained from plants [9]. The usage of plant based pharmaceuticals, such as opium, aspirin, digitalis, and quinine, have a long history in herbal remedies [8]. Some plants are used to cure one specific disease, whereas other plants are used in different circumstances. In the field of pharmacology, wild flora is very important and used in the production of new medicines as well as it provides immunity against many illnesses [9, 10].

Plants are not only used for medicinal purpose but also reflect the economic status for some indigenous peoples. The use of medicinal plants is growing rapidly and is estimated to reach the value of 5 trillion dollars (US) by 2050 [11]. The world’s population is expected to increase up to 10 billion by 2050 [12]. While the plant biodiversity is threatened by a variety of factors, including the increasing human population, climate change and anthropogenic factors are the major reasons of the loss of biodiversity [13]. According to the United Nation, more than one million species are at risk of extinction globally [14]. The woody flora is important to maintain the terrestrial ecosystem, conservation of water, prevent soil erosion, avoid floods and droughts, clean air, and water resources [15]. Local knowledge plays an important role in resource management, understanding and conserving antient practices, and play a vital role in saving the resources [14, 16]. Quantitative studies are very helpful to plan strategies for the conservation of natural plant resources [17, 18].

In Pakistan traditional medicine could have played an important role in providing health care to population [13, 19]. Only 12% medicinal plants are used for treatment of different diseases. The medicinal herbs are utilized for the cure of both animal and human diseases. Due to industrialization, over population and extensive collection, particular medicinal plant are near to extinction [20]. Peoples that are living in or near the forests are more dependent on forests than others and have more knowledge about the utilization of plants for various purposes [21]. The local communities living in Pakistan mostly use herbal remedies for treatment of different diseases [5]. The common diseases such as fever, cold, cough and diarrhea could be treated by locally available herbal teas and herbal powders and they have no side effects. Even today various locally produced drugs are still being used as remedies for different ailments [22]. Almost 40000–50000 local hakims are utilizing 200 medicinal plants in local recipes for the treatment of many ailments [20] and ethnobotanical knowledge on 600 plant species has been documented [23].

The folk and local healthcare knowledge has been passed orally from one generation to another instead of in the form of written document due to this reason the traditional knowledge is decreasing gradually [24]. There is a need to save this important conventional knowledge [23]. Therefore, the purpose of this study was to collect ethnobotanical data about local plants from the peoples of Mandi Ahmad Abad which may help and find new leads to collect raw material for drug discovery. We also aimed to compare local ethnobotanical data between our area of study and other areas of Pakistan as well as neighboring countries via the technique of Jaccard’s Similarity Index.

## Materials and methods

### Study area

The city Mandi Ahmad Abad, District Okara Pakistan was selected for collection of ethnobotanical data. This city shares boundary with India therefore its geographical importance for defense is high.

It was previously called Mandi Hira Singh and renamed in 1993 by the Government of the Punjab in respect for the services of Mirza Ahmad Baig famous local politician. It is a union council, an administrative subdivision of Depalpur Tehsil. It is situated between 30.65° N north latitude, 74.031° E longitude. It has a subtropical climate with annual average precipitation 200 mm and 24.5°C. The hottest months are May and June with maximum and minimum temperature 44°C and 2°C, respectively.

### Ethnobotanical survey

The most of available literature of ethnobotanical data was studied. To collect maximum information about local uses of plants, many ethnobotanical surveys were carried out from October, 2019 to April, 2020 in the area of Mandi Ahmad Abad. The ethnobotanical data was collected by providing semi-structured questionnaires and oral interviews. Interviews were taken from both males and females in fields, streets, homes and shops. Review Committee for Biomedical Research, University of Veterinary and Animal Sciences, Lahore, Pakistan approved the conduction of this study. Oral consent was obtained from participants before starting study. The interview from female was a difficult task because they were not allowed to talk with unknown persons. Only 34 females with the help of local inhabitants on special request were interviewed. Total 94 informants ranging from 15–75 years including males, females, farmers, hakims, shepherds, herdsmen, school boys and others have sound local knowledge about different uses of plants. Out of 94 informants, 60 were males and 34 were females. Different age groups of informants were made e.g. 15–25, 25–35, 35–45, 45–55, 55–65, and 65–75. The questionnaire was prepared in such a way to collect maximum data about different plants, including (a) name of informants, gender, age, job and qualification (b) information about plants e.g. local name of plant, parts used, method of preparation of recipe, mode of administration and ethnobotanical uses. Information about local uses of plants like food, fodder, fuel, timber, medicine, furniture and other uses was also collected [25]. The location of plants was recorded by taking quadrants by using GPS essentials application. A total 94 informants were interviewed and information regarding to their gender, marital status, age group, literacy level and socio-economics is given in the (Table 1).

**Table 1:** Demographic data of informants.

Categories	Number	Percentage	Education level	Number	Percentage
Gender			Illiterate	8	8.51
Men	60	63.83	Primary	15	15.96
Women	34	36.17	Middle	19	20.21
Total	94		Matric	23	24.47
**Socio-economics**	**Number**	**Percentage**	Intermediate	15	15.96
Farmers	44	46.81	Graduate	14	14.89
House wives	17	18.09	**Age group**	**Number**	**Percentage**
Shepherds	13	13.83	15–25	5	5.32
Teachers	3	3.19	25–35	9	9.57
Homeopathy doctors	2	2.13	35–45	13	13.83
Local Healers	6	6.38	45–55	19	20.21
Nurses	2	2.13	55–65	31	32.98
Shopkeepers	7	7.45	65–75	17	18.09
Total	94		Total	94	

### Collection and identification

Plants used by indigenous people and herbalists were collected from the study area. Samples of grasses, herbs, shrubs and trees were taken, dried, mounted on herbarium sheets and properly identified by using Flora of Pakistan [26]. Ethnobotanical data from local people was collected by providing semi-structured questionnaire, group meetings and interviews.

### Data analysis

The medicinal plants collected and identified from study area were organized in a table according to botanical names in alphabetical order, common names, family, parts used, rout of application and ethnobotanical uses. The accuracy and perfection of collected ethnobotanical data were checked and use value (UV), frequency of citation (FC), relative frequency citation index (RFCi), informant consensus factor (ICF) and Jaccard index (JI) by determined using different statistical tools.

#### Frequency citation (FC)

The information provided by informants for a specific plant with respect to local medicinal value was considered as frequency citation.

#### Relative frequency citation index (RFCi)

The value is calculated by dividing frequency of citation (FC) with total number of informants participating in a survey [27].

#### Use value (UV)

The relative importance of plants collected from study area was calculated by given formula;

$$UVi=\sum \frac{Ui}{Ni}$$

Here, Ui = Number of use report for specific plant by each informant

Ni = Number of total informants interviewed for specific plant.

#### Informant consensus factor

The informant consensus factor (FIC) based on the reported remedies was calculated for the various remedies using the formula [28];

$$FIC=\frac{Nur-Nt}{Nur-1}$$

Here,

Nur: is the number of used citation in each category

Nt: is the number of species used for particular ailment

#### Family importance value

The family Importance value (sum of all the use values of species in a family), and/or average family importance value (use values of all spp. in a family/number of species in the same family) was also determined.

#### Relative importance

It was calculated according to Bennett and Prance (2000);

RI=(BS+PH)*50

Where, BS is the normalized number of the body systems for which the species used and PH is the normalized number of the pharmacological properties or particular minor uses of the same species.

#### Jaccard index (JI)

The JI was calculated by comparison of previously published studies from other areas by analyzing the percentage of quoted species and their medicinal uses by using the following formula [29];

$$JI=\frac{C}{\left(A+B-C\right)}\times 100$$

“A” is the number of species of the area A, “B” is the number of species of the area B, “C” is the number of species common to both areas A and B.

In the present study, we calculated similarity index between our ethnobotanical survey and other studies which were carried out in different regions of Pakistan and neighboring countries.

## Results and discussion

The results of the present work are summarized below:

### Demographic information

The ethnobotanical data showed that the younger generation had less knowledge about the use of local plants compared to people aged 35 years and over, who had the most knowledge (Table 1). During the survey, most of the information was gathered from the male group (63.83%) compared to the female group (36.17%). The majority of knowledge was collected from the age group 55–65 years old (32.98%) and the minimum information was collected from the 20–25 year age group (5.32%). The ethnobotanical knowledge also varied according to the educational level of the community. The people who did matriculation (24.47%) had considerably more knowledge about indigenous plant usage than the graduate group (14.89%). The illiterate community of the study area had the least information about the plants (8.51%). The farmers of Mandi Ahmad Abad provided more ethnobotanical data for the plants (46.81%) followed by housewives (18.09%), shepherds (13.83%), shopkeepers (7.45%), local healers (6.38%), teachers (3.19%), homeopathic doctors (2.13%), and nurses (2.13%). Most of the population relied upon allopathic medicines and the modern health care system but the illiterate and less educated indigenous peoples predominantly used local medicinal plants to cure various ailments. As the modern health care system is growing and literacy levels are increasing, the indigenous knowledge is decreasing because the younger generation does not pay attention to this knowledge. The other studies reported that medicinal plant use is generally transmitted through the generations, but the older generation has been unable to impart traditional knowledge to the young, leading to a loss of information about biodiversity [30]. A study conducted in Bangladesh revealed the knowledge of medicinal plants was highest in the age group of 30–40 and lowest for the group aged 60 years and older [31].

### Diversity of local plants

The results showed that the study area is rich in useful plants (Table 2). It is an agricultural area and diversified with medicinal flora that is used by indigenous people to cure diseases and is also used for many other purposes. A total of 126 local plants belonging to 52 families were reported where Poaceae (13 spp.) was the predominant family followed by Leguminosae (12 spp.) and Solanaceae, Cucurbitaceae (10 spp. each) (Fig 1).

**Fig 1:** Contributions of top 12 families in ethnobotanical flora of Mandi Ahmad Abad.

**Table 2:** List of plants used in preparation of herbal formulation in the study area.

#	Botanical Name & Voucher No.	Local Name	Family	Parts used	Mode of administration	Recipes & Ethnobotanical use	FC	RFC	UV	RI
**1**	*Abelmoschus esculentus* (L.) Moench (ADN-701)	Bhindi	Malvaceae	Fruit	Oral	Fresh fruit is cooked as vegetable, and raw eating cure joint pain.	7.45	0.58	0.1	36.67
**2**	*Acacia nilotica* (L.) Delile (ADN-702)	Keekar	Leguminosae	Flower, Bean, Stem	Oral	About 10gm of flowers are soaked in 250 ml of water for 12 hours, filtered and drink to cure Leucorrhea. The dried bean powder (2 table spoons daily) is used for few days to relief backache. The boiled and dried beans are also used in pickles. The wood is utilized to make furniture, and as fuel wood.	11.7	0.92	0.17	55.00
**3**	*Achyranthus aspera* L. (ADN-703)	Puthkand/ Char chita	Amaranthaceae	Whole plant	Oral	The powder is used for treatment of cough and kidney problems	2.13	0.17	0.03	36.67
**4**	*Albizia procera* (Roxb.) Benth (ADN-704)	Shirin	Leguminosae	Bean, Seed, Leaves	Oral	The dried beans and seeds powder (1/2 tea spoon) with water 3 times in a day to cure piles. Fresh Leaves are used for fodder.	5.32	0.42	0.07	36.67
**5**	*Alhagi maurorum* Medik. (ADN-716)	Jawaiyan	Leguminosae	Whole plant	Oral	The powder is used in medicines to cure diseases of reproductive system.	1.06	0.08	0.01	18.33
**6**	*Allium cepa* L. (ADN-705)	piyaz	Amaryllidaceae	Bulb	Oral	The fresh bulb is used for blood purification, to enhance maleness, as salad and cooking purpose.	9.57	0.75	0.18	55.00
**7**	*Allium sativum* L. (ADN-706)	Lehsan	Amaryllidaceae	Bulb	Oral	The fresh bulbs are used to control blood pressure, do blood purification, and in cooking, chutney and pickles.	8.51	0.67	0.16	45.00
**8**	*Aloe vera* (L.) Burm.f. (ADN-707)	Kawar gandal	Xhanthorrhoeaceae	Whole plant	Oral, Topical	The mucilaginous pulp is orally used as anti-constipatory, backache and proper functioning of liver. Pulp is directly applied on skin for whitening of skin and other skin disorders.	9.57	0.75	0.14	73.33
**9**	*Amaranthus viridus* L. (ADN-708)	Chulai	Amaranthaceae	Shoot	Oral	The shoot is cooked as vegetable to cure constipation, and kidney stones. Fresh aerial parts are used as fodder for livestock.	7.45	0.58	0.14	63.33
**10**	*Anagallis arvensis* L. (ADN-709)	Billi booti	Primulaceae	Aerial part	Oral	Fresh aerial parts are used as fodder for livestock.	3.19	0.25	0.03	18.33
**11**	*Andropogan sorghum* L. (ADN-710)	Jawar	Poaceae	Aerial part	Oral	Fresh aerial parts are used as fodder for livestock.	5.32	0.42	0.05	18.33
**12**	*Arundo donax* L. (ADN-711)	Naryan	Poaceae	Root, Whole plant	Topical	Poultice of roots applied on forehead for headache. Dried plants used in making roofs of huts.	4.26	0.33	0.07	26.67
**13**	*Avena sativa* L. (ADN-712)	jai	Poaceae	Seed	Oral	The powder dried seeds mixed with water for stomach disorders.	6.38	0.5	0.06	18.33
**14**	*Azadirachta indica* A. Juss. (ADN-713)	Neem	Meliaceae	Fruit, Seed, Aerial parts	Oral	The infusion or syrup from fruit and seeds used for diabetes, blood purifier, for pustules and pimples. Brush of branches is used for tooth cleaning.	12.77	1	0.22	73.33
**15**	*Bauhinia variegata* L. (ADN-714)	Kachnaar	Leguminosae	Flower	Oral	The powder dried flowers (1 tea spoon) or water extract for normal blood pressure and stomach disorders. Fresh flowers are cooked as a vegetable.	6.38	0.5	0.1	55.00
**16**	*Bennincasa cerifera* (Thunb) ADN-715	Petha	Cucurbitaceae	Fruit	Oral	Fruit is cooked as a vegetable.	4.26	0.33	0.04	18.33
**17**	*Bombax ceiba* L. (ADN-717)	Sumbal	Malvaceae	Root, Latex, Stem	Oral	The infusion of roots in water for proper functions of male reproductive systems. The latex orally taken with water for menstrual problems. Wood is used for sheets formation.	5.32	0.42	0.1	45.00
**18**	*Bombosa arundinosa* (Retz.) ADN-718	Bans	Poaceae	Stem	Oral	Water extract is used for asthma. Dried plants are used for making huts, building materials and fuel	7.45	0.58	0.11	36.67
**19**	*Bougainvillea berberidifolia* Heimerl. (ADN-719)	Bougainvillea	Nyctaginaceae	Leaves	Oral	Extract of leaves use daily to control worms of abdomen.	2.13	0.17	0.02	18.33
**20**	*Brassica oleracea* L. var. *capitata* (ADN-722)	Band gobhi	Brassicaceae	Aerial part	Oral	Cooked as vegetable and also used as salad and fodder.	5.32	0.42	0.11	35.00
**21**	*Brassica oleracea* Lam. var. *botrytis* (ADN-723)	Phool gobhi	Brassicaceae	Aerial part	Oral	Cooked as vegetable, and used as fodder for animals.	7.45	0.58	0.13	26.67
**22**	*Brassica rapa* subsp. *rapa* L. (ADN-721)	Shaljam	Brassicaceae	Root, Leaves	Oral	Roots are cooked as vegetables, generate blood and improve digestion. Leaves are also used as fodder.	7.45	0.58	0.14	63.33
**23**	*Brassica rapa var*. *campestris* L. (ADN-720)	saag	Brassicaceae	Seeds, Aerial parts	Oral	Seeds are used for oil extraction. After oil extraction, the residue called "khall" is formed used for livestock for increasing milk production. Fresh leaves cooked as a vegetable and fresh leaves directly used as a fodder.	8.51	0.67	0.22	53.33
**24**	*Bryophyllum pinnatum* (Lam.) Oken (ADN-724)	Pathar chat	Crassulaceae	Leaves	Oral	Water extract or dried powder of leaves to cure kidney stones.	4.26	0.33	0.04	18.33
**25**	*Calotropis procera* (Aiton) Dryand. (ADN-725)	Akk	Apocynaceae	Leaves, Flower, Latex	Topical	Leaves are mixed with oil and heat to get infusion for joints pain. Flowers or latex directly used to cure wounds, psoriasis and snake bite.	6.38	0.5	0.12	55.00
**26**	*Cannabis sativa* L. (ADN-726)	Bhung	Cynnabaceae	Seeds, Leaves	Oral	Seeds are orally taken with water as a Anti-cancerous and used in infertility of females. Dried leaves used in narcotics.	8.51	0.67	0.12	45.00
**27**	*Capsicum annum* L. (ADN-727)	Shimla mirch	Solanaceae	Fruit	Oral	Fruit is used as a vegetable.	2.13	0.17	0.02	18.33
**28**	*Capsicum frustescens* L. (ADN-728)	Sabz mirch	Solanaceae	Fruit, Seeds	Oral	Seeds used in fever, fruit are used in chutney, pickle and cooking purpose.	9.57	0.75	0.15	26.67
**29**	*Cassia fistula* L. (ADN-729)	Amaltas	Leguminosae	Seeds	Oral	The powder of seeds used in stomach disorders.	3.19	0.25	0.03	18.33
**30**	*Chenopodium album* L. (ADN-730)	Bathu	Amaranthaceae	Leaves	Oral	Leaves cooked separately or mixed with brassica for normal blood pressure, Anti-constipatory and vegetable for humans.	8.51	0.67	0.14	55.00
**31**	*Chenopodium murale* L. (ADN-731)	krund	Amaranthaceae	Aerial Part	Oral	The decoction of leaves is orally used for pustules, pimples and wounds. Aerial parts are used as fodder.	5.32	0.42	0.07	36.67
**32**	*Cicer arietinum* L. (ADN-732)	channy	Leguminosae	Seeds, leaves	Oral	The powder of seeds used for diabetes, for weak eye sight and proper functioning of stomach. The leaves of young plants used as vegetable for humans and fodder for animals.	11.7	0.92	0.16	55.00
**33**	*Cichorium intybus* L. (ADN-733)	Kaasni	Compositae	Whole plant	Oral	Syrup preparation to cure hepatitis, jaundice and proper functioning of liver. Decoction or water extract by grinding the parts of plant used for blood purification.	5.32	0.42	0.15	63.33
**34**	*Citrullus colocynthis* (L.) Schrad (ADN-734)	Korh tumba	Cucurbitaceae	Fruit, Leaves	Oral	Powder used as anti-constipatoty, to cure Asthma, for stomach disorders and rheumatism. Leaves are used as fodder.	4.26	0.33	0.11	81.67
**35**	*Citrullus lanatus* (Thunb.) Matsum. & Nakai (ADN-735)	Tarbooz	Cucurbitaceae	Fruit	Oral	Fruit is used as a food, for proper liver functioning and to increase blood production.	6.38	0.5	0.09	36.67
**36**	*Citrus limon* (L.) Osbeck (ADN-737)	Leemo	Rutaceae	Fruit	Oral, Topical	Fruit juice is used to make drink “askanjbeen” and used as anti-vomiting, to cure stomach disorders and pickle formation. The extract of fruit is directly applied on skin for cleaning.	7.45	0.58	0.12	63.33
**37**	*Convolvulus arvensis* L. (ADN-738)	Valoor	Convolvulaceae	Whole plant	Oral	Grind and separate its extract and use (1 Tea spoon daily) for worms of stomach. Whole plant is used for treatment of dysentery in goats and sheep.	4.26	0.33	0.05	26.67
**38**	*Cordia myxa* L. 9ADN-739)	Lasoorha	Boraginaceae	Fruit	Oral	Fruit is directly edible and used for treatment of ulcer of stomach, joints pain and body’s weakness. Fried fruit used in pickle formation.	6.38	0.5	0.11	63.33
**39**	*Cordia sinensis* Lam. (ADN-740)	Goondi	Boraginaceae	Fruit	Oral	Fruit is edible, and cure stomach inflammation, cough, throat and joints pain. Leaves are used as fodder.	5.32	0.42	0.1	63.33
**40**	*Coriandrum sativum* L. (ADN-741)	Dhania	Apiaceae	Leaves	Oral	The powder of seeds used in condiments. Leaves are used in chutney and other cooked dishes	5.32	0.42	0.05	18.33
**41**	*Cucumis melo* L. (ADN-742)	Kharbooza	Cucurbitaceae	Seeds, Pericarp	Oral	The powder of dried seeds and pericarp mix with honey to make tablets to cure kidney stones. Fruit is used in fever and as a food.	4.26	0.33	0.05	36.67
**42**	*Cucumis melo* var. *agrestis* Naudin (ADN-743)	Chibbar	Cucurbitaceae	Whole plant	Oral	Fruit is edible. Powder of fruit is used in stomach disorders and skin problems. The leaves are used as a fodder.	8.51	0.67	0.12	63.33
**43**	*Cucumis sativus* L. (ADN-744)	Kheera	Cucurbitaceae	Fruit	Oral	Fruit is used for proper functioning of stomach and digestion of food.	4.26	0.33	0.05	36.67
**44**	*Cucurbita pepo* L. (ADN-745)	Kaddo	Cucurbitaceae	Fruit	Oral	Fruit is used as a vegetable and efficient working of stomach.	5.32	0.42	0.07	36.67
**45**	*Curcuma longa* L. (ADN-746)	Haldi	Zingiberaceae	Rhizome	Oral	The powder of rhizome is used for joints pain and in condiments.	5.32	0.42	0.09	36.67
**46**	*Cuscuta reflexa* Roxb. (ADN-747)	Amar bail	Convolvulaceae	Whole plant	Oral	Infusion in oil and tonic formation for efficient growth of hairs, anti-lice and anti-dandruff. Cooked juice for flu and influenza.	8.51	0.67	0.1	26.67
**47**	*Cynodon dactylon* (L.) Pers. (ADN-748)	Khabal ghaas	Poaceae	Whole plant	Topical	Poultice/ paste are applied on wounds and skin infections.	2.13	0.17	0.02	18.33
**48**	*Dalbergia sissoo* DC. (ADN-749)	Sheesham	Leguminosae	Leaves, Bark, Beans, Stem	Oral	Infusion in water for proper functioning of male reproductive system. Wood is used in furniture and fuel.	6.38	0.5	0.1	36.67
**49**	*Datura innoxia* Mill. (ADN-750)	Dhatoora	Solanaceae	Seeds	Oral, Topical	Directly used or taken in powder form to cure scabies, pimples and other skin problems.	5.32	0.42	0.06	35.00
**50**	*Daucus carota* L. (ADN-751)	Gajar	Apiaceae	Root	Oral	Root is used or cooked as a vegetable, generates blood and used in making salad.	7.45	0.58	0.13	45.00
**51**	*Desmostachya bipinnata* (L.) Stapf (ADN-752)	Dub ghaas	Poaceae	Whole plant	Oral	Decoction is used for the treatment of fever and headache.	2.13	0.17	0.03	26.67
**52**	*Eclipta prostrata* (L.) L. (ADN-753)	Bhangra	Compositae	Whole plant	Oral	Powder dried parts of plants is used for tooth cleaning.	1.06	0.08	0.01	18.33
**53**	*Eucalyptus camaldulensis* Dehnh. (ADN-754)	sufaida	Myrtaceae	Whole plant, Stem	Oral	Fresh parts or powder is used to cure flu and influenza. Wood is used for fuel, timber and furniture.	12.77	1	0.16	26.67
**54**	*Euphorbia granulata* Forssk. (ADN-816)	Hazar dani	Euphorbiaceae	Whole plant	Oral	Powder is used for treatment of dysentery.	1.06	0.08	0.01	18.33
**55**	*Ficus benghalensis* L. (ADN-755)	Bohr	Moraceae	Whole plant, Aerial roots, Latex	Oral	The powder of aerial roots used for proper function of liver and blood production. Syrup from whole parts of plant is used to cure asthma. Latex is mixed with its bark used in the treatment of gonorrhea and for proper function of male reproductive system.	9.57	0.75	0.13	81.67
**56**	*Ficus religiosa* L. (ADN-756)	Peepal	Moraceae	Bark, Fruit, Latex	Oral	The powdered of dried bark is used for tooth cleaning. The cooked juice of bark is used as anti-vomiting. The powder of bark mixed with latex used for treatment of gonorrhea. The powder of bark, fruit and latex is used to relief from body pain.	7.45	0.58	0.13	71.67
**57**	*Foeniculum vulgare* Mill. (ADN-757)	Sounf	Apiaceae	Seeds	Oral	The powder of seeds mixed with sugar (2 tea spoon) for weakness of eyesight and stomach disorders.	6.38	0.5	0.09	36.67
**58**	*Fragaria ananassa* (Duchesne ex Weston) Duchesne ex Rozier (ADN-758)	Strawberry	Rosaceae	Fruit	Oral	Fruit is edible and generates blood and full with iron.	3.19	0.25	0.03	18.33
**59**	*Fumaria indica* (Hausskn.) Pugsley (ADN-759)	Pit papra	Papaveraceae	Whole plant	Oral	Syrup preparation by boiling and adding sugar for allergy and scabies.	2.13	0.17	0.02	18.33
**60**	*Gossypium arboreum* L. (ADN-760)	Kapas	Malvaceae	Leaves, Seeds, Flowers, Stem	Oral	Water extract of leaves is used in medicines for regular menstrual cycle. Seeds are used for oil extraction, cotton and banoola is also obtained used as a fodder for animals. Dried stem is used as a fuel.	8.51	0.67	0.14	53.33
**61**	*Hibiscus rosa-sinensis* L. (ADN-761)	Shoe flower	Malvaceae	Flowers	Oral	Syrup formation from fresh or dried flowers used to cure heart diseases.	1.06	0.08	0.01	18.33
**62**	*Hordeum vulgare* L. (ADN-762)	Jou	Poaceae	Seeds	Oral	The powder of seeds is used for making breads and proper activity of stomach. Fresh aerial parts of plant are used as a fodder.	6.38	0.5	0.1	36.67
**63**	*Ipomeoe cairica* (L.) ADN-763	Ishq peecha	Convolvulaceae	Seeds	Oral	Seeds orally taken with water used in medicines for normal working of male reproductive system	3.19	0.25	0.03	18.33
**64**	*Jasminum sambac* (L.) Aiton (ADN-764)	Chambaili	Oleaceae	Whole plant	Nil	Grown in lawns and parks having ornamental value.	5.32	0.42	0.07	26.67
**65**	*Lawsonia inermis* L. (ADN-765)	Mehndi	Lythraceae	Leaves	Topical	Paste of dried leaves or powder used in feet burning, to color hands, feet and hairs.	6.38	0.5	0.06	26.67
**66**	*Lepidium didymum* L. (ADN-766)	Afsanteen	Brassicaceae	Leaves	Oral	Decoction from fresh leaves for scabies, blood purifier and liver problems. Flowers orally taken with water for the treatment of diabetes.	8.51	0.67	0.17	81.67
**67**	*Luffa cylindrica* (L.) M.Roem. (ADN-767)	Toori	Cucurbitaceae	Fruit	Oral	Cooked fruit used as a vegetable.	4.26	0.33	0.04	18.33
**68**	*Lycopersicon esculentum* Mill. (ADN-768)	Tamatar	Solanaceae	Fruit	Oral	Fruit is used for blood production, used in salad and cooking purpose	5.32	0.42	0.1	45.00
**69**	*Malva parviflora* L. (ADN-769)	Chiri choga	Malvaceae	Leaves	Oral	Leaves decoction is used to cure stomach disorders.	4.26	0.33	0.04	18.33
**70**	*Mangifera indica* L. (ADN-770)	Aam	Anacardiaceae	Fruit, Seeds	Oral	The powder of seeds (1–2 tea spoons) helpful in the treatment of leucorrhea. Fruit is edible and increase production of blood, pickle, chutney and marmalade.	8.51	0.67	0.12	55.00
**71**	*Melia azedarch* L. (ADN-771)	bakaen	Meliaceae	Fruit, Stem	Oral	Grind fruits and mixed with animal’s fodder for efficient digestion and more milk production In livestock. Fruit is edible and function as a blood purifier. Wood is used for fuel and furniture.	6.38	0.5	0.1	73.33
**72**	*Melilotus indica* (L.) All. (ADN-772)	Sainjhi	Fabaceae	Whole plant, Seeds	Oral	Dried powder of seeds used for proper bowel functions. Aerial parts are used as a fodder	4.26	0.33	0.07	45.00
**73**	*Mentha arvensis* L. (ADN-773)	Podina	Lamiaceae	Whole plant	Oral	Powder, paste or extract for stomach acidity and chest burning.	6.38	0.5	0.09	26.67
**74**	*Mentha longifolia* (L.) L. (ADN-774)	Jangli podina	Lamiaceae	Whole plant	Oral	Grind by using pestle & mortar, and squeeze the juice, taken orally to cure piles, stomach disorders and blood purification.	7.45	0.58	0.1	45.00
**75**	*Momordica charantia* L. (ADN-775)	Kareela	Cucurbitaceae	Fruit, Pericarp	Oral	Fruit with its covering place in water whole night and drink water in morning for diabetes, allergy and pustules.	8.51	0.67	0.12	45.00
**76**	*Moringa oleifera* Lam. (ADN-776)	Suhanjna	Moringaceae	Beans, Leaves	Oral	The powder of leaves (2 tea spoon daily) used to cure diabetes, backbone pain, eye sight weakness. Beans are cooked, and used as food and in pickle formation. Leaves are used as a fodder for increasing milk and meat production for livestock.	6.38	0.5	0.15	81.67
**77**	*Morus alba* L. (ADN-777)	Sufaid shahtoot	Moraceae	Fruit, Stem	Oral	Fresh or dried fruit is edible and used to cure inflammation of throat and problems associated with respiratory tract. Wood is used for fuel, timber and furniture.	10.64	0.83	0.16	45.00
**78**	*Morus nigra* L. (ADN-778)	Kala shahtoot	Moraceae	Fruit, Leaves	Oral	Fresh, dried or syrup of fruit is used for treatment of cough, respiratory tract infection and worms of abdomen. Leaves are used as a fodder for livestock.	9.57	0.75	0.14	55.00
**79**	*Musa paradisiaca* L. (ADN-779)	Kela	Musaceae	Fruit, Stem	Oral	Fresh fruit is edible used to cure diarrhea and increasing body weight. Water extract from stem is used in the treatment of leucorrhea.	6.38	0.5	0.11	55.00
**80**	*Nicotiana tabacum* L. (ADN-780)	Tobacco	Solanaceae	Leaves	Oral	Dried and crushed leaves are used in cigarette. Water extract from leaves is used as an antiseptic.	4.26	0.33	0.06	26.67
**81**	*Ocimum basilicum* L. (ADN-821)	Tulsi	Lamiaceae	Seeds, Leaves	Oral	Water soaked seeds drink with water used for urinary tract infection and reduce swelling. Cooked juice of leaves used to cure cough, flu and other respiratory infections.	5.32	0.42	0.1	63.33
**82**	*Oryza sativa* L. (ADN-781)	Chawal	Poaceae	Seeds, Stem	Oral	Cooked seeds and powder of seeds used as a food for humans. Dried stem used as fuel.	3.19	0.25	0.04	18.33
**83**	*Oxalis corniculata* L. (ADN-782)	Torshuk	Oxalidaceae	Leaves	Oral	Leaves are grounded to paste, followed by juice extraction and taken to treat stomach and liver dis-functioning.	5.32	0.42	0.07	36.67
**84**	*Peganum harmala* L. (ADN-783)	Harmal	Nitrariaceae	Seeds	Oral	The powder of seed (1 tea spoon) is used for diabetic patients and joints pain.	3.19	0.25	0.05	36.67
**85**	*Pennisetum glaucum* (L.) R.Br. (ADN-784)	Bajrah	Poaceae	Seeds, Stem	Oral	The powder of seeds used to cure joints pain. Stem is used as a fodder.	4.26	0.33	0.06	36.67
**86**	*Pentatropis nivalis* (J.F.Gmel.) D.V.Field & J.R.I.Wood (ADN-785)	Fareed	Apocynaceae	Leaves	Oral	Leaves paste mixed with honey is taken to regulate and correct menstrual cycle.	2.13	0.17	0.02	18.33
**87**	*Phalaris minor* Retz. (ADN-786)	Dumbi sitti	Poaceae	Aerial part	Oral	Aerial parts are used as a fodder for animals.	4.26	0.33	0.04	18.33
**88**	*Phoenix dactylifera* L. (ADN-787)	Khajoor	Arecaceae	Fruit	Oral	Fruit is edible and improves digestion, provide strength to body.	7.45	0.58	0.1	36.67
**89**	*Phylla nodiflora* L. (ADN-788)	Gandh booti	Verbenaceae	Leaves	Oral	Leaves are used as a fodder for livestock.	3.19	0.25	0.03	18.33
**90**	*Pisum sativum* L. (ADN-789)	Matar	Leguminosae	Beans, Aerial parts	Oral	Seeds are used as vegetable. Aerial parts are used as fodder.	7.45	0.58	0.1	26.67
**91**	*Polygonum aviculare* L. (ADN-791)	Hind ki raani	Polygonaceae	Whole plant	Oral	Infusion from dried plant orally taken to cure leucoderma or vitiligo.	2.13	0.17	0.02	18.33
**92**	*Pongamia pinnata* (L.) Pierre (ADN-790)	Sukh chain	Leguminosae	Aerial parts, Leaves	Oral	The branches are used for cleaning tooth. Leaves are used as a fodder.	5.32	0.42	0.06	36.67
**93**	*Populas nigra* L. (ADN-792)	Paplar	Salicaceae	Bark, Fruit	Oral	The powder from bark and fruit used for treatment of arthritis and backache.	6.38	0.5	0.07	26.67
**94**	*Portulaca oleracea* L. (ADN-793)	Qulfah	Portulacaceae	Whole plant	Oral	Powder or boiled whole plant in water and orally taken to cure constipation, jaundice and skin problems.	4.26	0.33	0.06	55.00
**95**	*Praecitrullus fistulosus* (Stocks) Pangalo (ADN-736)	Tenda	Cucurbitaceae	Fruit	Oral	Fruit is used as a vegetable.	4.26	0.33	0.04	18.33
**96**	*Prosopis juliflora* (Sw.) DC. (ADN-794)	Pahari keekar	Leguminosae	Beans, Stem	Oral	Fresh or dried beans used as a fodder for goats. Wood is used as fuel.	2.13	0.17	0.04	26.67
**97**	*Prunus persica* (L.) Batsch (ADN-795)	Desi aaro	Rosaceae	Fruit, Leaves	Oral	Fresh or dried fruit is edible for diabetes, proper functioning of stomach and worms of abdomen, Leaves are used as a fodder.	6.38	0.5	0.11	63.33
**98**	*Psidium guajava* L. (ADN-796)	Amrood	Myrtaceae	Leaves, Fruit	Oral	The decoction or cooked juice of leaves for diabetes, proper functioning of stomach And toothache. Fruit is edible and anti-constipatory.	8.51	0.67	0.14	53.33
**99**	*Punica granatum* L. (ADN-797)	Anaar	Lythraceae	Fruit	Oral	Fruit is edible generates blood and used for normal activity of stomach.	6.38	0.5	0.09	36.67
**100**	*Raphanus raphanistrum* subsp. *sativus* (L.) Domin (ADN-798)	Mooli	Brassicaceae	Root, Leaves	Oral	Root is used or cooked as a vegetable, proper functioning of stomach and used in salad. Leaves are used as a fodder.	7.45	0.58	0.14	53.33
**101**	*Ricinus communis* L. (ADN-799)	Arind	Euphorbiaceae	Seeds, Fruit	Oral, Topical	Oil extract from seeds used in medicines of rheumatism and arthritis and prevention of pregnancy.	5.32	0.42	0.09	55.00
**102**	*Rosa alba* L. (ADN-800)	Chitta gulab	Rosaceae	Whole plant, Flower	Topical	Water extract of flowers used to cure eyes infection. Whole plant have ornamental value.	4.26	0.33	0.06	36.67
**103**	*Rosa indica* L. (ADN-801)	Lal gulab	Rosaceae	Flower	Oral, Topical	Flower petals mixed with sugar are used in making “Gulkand” for stomach disorders in humans and increasing milk production in livestock. Water extract of flowers is used for eyes infection, softness of skin. Whole plant has ornamental value.	11.7	0.92	0.18	91.67
**104**	*Rumex dentatus* L. (ADN-802)	Jangli palak	Polygonaceae	Seeds, Leaves	Oral	The powder of seeds and leaves or directly used for normal working of genital organs. Leaves are used as a fodder for animals.	4.26	0.33	0.05	36.67
**105**	*Saccharum officinarum* L. (ADN-803)	Ganna	Poaceae	Stem	Oral	The stem juice is concentrated by boiling to local sweet called “Gurr”, Sugarcane juice is advised in case of liver and stomach disorders. Aerial parts are used as fodder.	8.51	0.67	0.17	71.67
**106**	*Salvadora oleoides* Decne. (ADN-804)	Ban	Salvadoraceae	Root	Oral	Fresh or dried roots are used as “miswak” or tooth-brush for tooth cleaning.	4.26	0.33	0.04	18.33
**107**	*Sesamum indicum* L. (ADN-805)	Til	Pedaliaceae	Seeds	Oral	Seeds are used for oil extraction and cure increased urination.	8.51	0.67	0.1	36.67
**108**	*Solanum americanum* Mill. (ADN-806)	peelak/ mako	Solanaceae	Whole plant, Fruit	Oral	Decoction from whole plant is used as a blood purifier to cure allergy and inflammation. Fruit is edible and used as anti-constipatory.	7.45	0.58	0.12	73.33
**109**	*Solanum melongena* L. (ADN-807)	Baingan	Solanaceae	Fruit	Oral	Cooked fruit is used for treatment of kidney stones and as a vegetable.	3.19	0.25	0.05	36.67
**110**	*Solanum tuberosum* L. (ADN-808)	Aloo	Solanaceae	Tuber, Stem	Oral	Tuber is edible and used as food. Stem is used as a fodder.	4.26	0.33	0.06	26.67
**111**	*Solanum virginianum* L. (ADN-809)	Bhatkari	Solanaceae	Whole plant	Topical	Whole plant boiled in water and wash infected area with this boiled water used as an Anti-inflammatory.	1.06	0.08	0.01	18.33
**112**	*Sonchus asper* (L.) Hill (ADN-810)	Bhattal/ Sonchal	Compositae	Leaves, Whole plant	Oral, Topical	Powder from whole dried plant applied on burns and wounds. Fresh leaves are used for fodder.	4.26	0.33	0.06	36.67
**113**	*Syzygium cumini* (L.) Skeels (ADN-811)	jaman	Myrtaceae	Whole plant, Seeds, Leaves	Oral	Decoction from whole plant is used to cure diarrhea, stomach disorders, proper liver functioning. The powder of seeds is used to cure diabetes and blood purification. Leaves are used as a fodder.	9.57	0.75	0.18	100.00
**114**	*Thuja occidentalis* L. (ADN-812)	Saro/ Mazoo	Cupressaceae	Seeds	Oral	The powder of seeds is used for strengthening of teeth and gums, egg production in females and poultry.	3.19	0.25	0.03	36.67
**115**	*Tinospora sinensis* (Lour.) Merr. (ADN-813)	Gloo	Menispermaceae	Whole plant	Oral	The powder of whole plant parts is used for treatment of typhoid and liver inflammation.	3.19	0.25	0.05	45.00
**116**	*Tithonia diversifolia* (Hemsl.) A.Gray (ADN-814)	Jangli gainda	Compositae	Seeds, Leaves	Oral	Seeds are orally taken with water for treatment of piles. Leaves used as fodder.	5.32	0.42	0.07	36.67
**117**	*Trianthema potulacastrum* L. (ADN-815)	It sit	Aizoaceae	Whole plant, Aerial parts	Oral	The juice is used to treat kidney stones.	5.32	0.42	0.01	36.67
**118**	*Tribulus terrestris* L. (ADN-817)	Bhakhra	Zygophyllaceae	Seeds, Aerial parts	Oral	The powder of seeds is used for kidney stones and backache. Aerial parts are used as a fodder.	6.38	0.5	0.09	55.00
**119**	*Trigonella foenum-graecum* L. (ADN-818)	Methi	Leguminosae	Whole plant	Oral	Powder from dried parts of plant is used for joints pain and blood purifier. Stem is cooked and use as vegetable.	7.45	0.58	0.12	55.00
**120**	*Triticum aestivum* L. (ADN-819)	Gandum	Poaceae	Fruit, Stem	Oral	The immature fruit is used to enhance milk production. “Tori” wheat straw is mixed with other fodder as animal feed.	5.32	0.42	0.07	26.67
**121**	*Typha elephantina* Roxb. (ADN-820)	Bora	Typhaceae	Stem	Nil	Dried stem is used in forming mats.	4.26	0.33	0.04	18.33
**122**	*Vigna radiata* (L.) R.Wilczek (ADN-822)	Moongi	Leguminosae	Beans, Stem	Oral	Cooked beans used as vegetable for humans and to cure joints pain.	4.26	0.33	0.05	36.67
**123**	*Vitis vinifera* L. (ADN-823)	Angoor	Vitaceae	Fruit, Stem	Oral	Fruit is edible and used for proper functioning of heart and generates blood. Extract of stem is used for treatment of jaundice.	5.32	0.42	0.09	45.00
**124**	*Withania somnifera* (L.) Dunal (ADN-824)	Iksan	Solanaceae	Whole plant	Oral, Topical	Infusion in oil or powder to cure Joints pain, arthritis, rheumatic disorders, pustules and pimples	3.19	0.25	0.04	45.00
**125**	*Zea mays* L. (ADN-825)	Makai	Poaceae	Seeds, Stem	Oral	Flour is used for making breads. Fresh stem used as fodder an dried stem used as fuel	6.38	0.5	0.07	26.67
**126**	*Ziziphus jujuba* Mill. (ADN-826)	Beri	Rhamnaceae	Fruit, Leaves, Stem	Oral	Fruit is edible for eye sight, proper hairs growth and joints pain. Leaves are used as fodder. Wood is used for fuel and furniture.	5.32	0.42	0.11	63.33

### Herbal therapies and preparation

More than 50 uses of plants were reported and many plant species were used against diseases including liver problems, skin disorders, heart problems, stomach disorders, respiratory tract infections and diabetes etc. A total of 25, 12 and 10 plant species were found effective against stomach disorders, joint pain and blood purification, respectively. Different parts of the local plants were used to prepare many local remedies. Among the different plant parts used, fruit were the favored part with (18.82%) usage in local remedies followed by leaves (18.28%) whole plant (16.13%), seeds (15.05%), stem (10.75%), aerial parts (6.99%), flowers (4.30%), roots (3.23%), latex (2.69%), bark (1.61%), bulb (1.08), tubers and rhizome (0.54%) (Fig 2). Different recipes were prepared from indigenous plant species i.e. infusion, decoction, powder, freshly cooked, cooked juice, poultice, porridge, water soaked seeds and infusion in oil etc. in the study area [32]. In these recipes, fresh herbs were used the most (22.5%) followed by powder (17.5%) and freshly cooked (11.3%) by local inhabitants. Flowers of *Acacia nilotica* were used for the treatment of leucorrhea, the bulb of *Allium sativum* is used to control blood pressure, Latex from *Bombax ceiba* is used to cure menstrual problems, seeds of *Cassia fistula* are used for stomach disorders, powder from *Citrullus colocynthis* is used for constipation and to cure asthma, the fruit of *Cordia myxa* is used to cure ulcers of the stomach and joint pain and fruit yielding plants provide a rich source of food but also provide numerous vitamins. Previous studies also reported the use of these plants against cure of different diseases [33–36].

**Fig 2:** Different parts of plants used by local people in herbal preparations.

### Mode of administration

Most of the herbal medicines are used orally by indigenous people but a few of the medicines are applied in the form of a paste or a poultice applied directly to the body (Table 2). The oral mode of ingestion is considered the best method for the treatment of different ailments but in skin disorders like skin allergies, wounds, pustules and pimples, herbal medicines are applied directly to the skin. Many plants of the same family or from different families were reported to be just as effective against a single disease [28].

### Relative importance of medicines

To evaluate the relative importance of indigenous plants, the use value was calculated for each plant. The result of this study tells us that *Azadirachta indica* shows a maximum use value (UV = 0.22) with a minimum use value (UV) indicated by *Alhagi maurorum*, *Eclipta prostrata*, *Hibiscus rosa-sinensis*, *Solanum virginianum* and *Trianthema potulacastrum* (UV = 0.01). It is clear from the formula sheet that the plant with the higher UV value is used in many more recipes for different purposes and the plants with the lower UV value are used in a more limited amount for the treatment of ailments across many other recipes.

### Informants consensus factor

The result of this study shows that hepatitis, ulcer of the stomach, bowel disorders, urinary problems, psoriasis, cancer, leucoderma, increased urination, antiseptic and burning feet were most prevalent in the study area with an ICF value (1.00). Followed by leucorrhea, which was second, with an ICF value (0.89) and vomiting was in third place, with an ICF value (0.86). Many other common diseases e.g., acidity of the stomach (ICF = 0.83), blood pressure (ICF = 0.82) and piles (ICF = 0.71) were observed with the calculation of the ICF value.

### Jaccard’s similarity index

Jaccard’s similarity index shows the degree of similarity related species cited between our study and other studies carried out in different areas of the world. The highest Jaccard’s similarity index value (JI = 0.329) shows that plant species reported in our study are more similar with [37] followed by [8] with Jaccard’s index value (JI = 0.283), and followed by [25] with Jaccard’s index value (JI = 0.245). The maximum Jaccard’s index value for uses comparison is (JI = 0.28) for study of [37], followed by (JI = 0.24) for [38] and Jaccard’s index value (JI = 0.24) for [25] was on third number. The highest Jaccard’s similarity index value shows the highest similarity between two studies of different areas.

## Conclusion

The current study reveals that the study area is diversified cereal, wild and many other medicinal plants. This is the first ethnobotanical survey of this study area. During this study very important information is collected with many medicinal plants. Reported medicinal plants are used to cure more than 50 ailments including heart diseases, respiratory tract infection, stomach disorders, hepatitis, joints pain and diabetes by indigenous people. Unfortunately, traditional knowledge about medicinal plants is decreasing day by day as young generation relies on allopathic medicines. Many people of this study area did not even know about ethnobotanical or medicinal uses of a single plant. The excessive use of medicinal plants, over grazing, deforestation and anthropogenic activities threatened the species. Most of the people are unaware from conservation strategies and this leads to the extinction of many species. On the basis of results of current survey, urgent attention is required for the conservation and documentation of traditional knowledge about plants and conservation of medicinal plants.

## Supporting information

S1 File Questionnaire for ethnobotanical survey of plants used by the people of Mandi Ahmad Abad, Okara. (PDF)

S2 File Excel data sheet for various ethnobotanical analyses. (XLSX)
